The article "Disseminated Tuberculosis Post COVID-19 Infection: A Case Report" was published in 2022. Journal: Cureus.

# Disseminated Tuberculosis Post COVID-19 Infection: A Case Report

**DOI:** 10.7759/cureus.31489

**Published:** 2022-11-14

**Authors:** Mohammed A Almatrafi, Khadeeja Awad, Nouf Alsahaf, Sarah Tayeb, Adil Alharthi, Nada Rabie, Rehab Fadag, Hassan Alwafi, Rayan Salawati, Aseel K Alhindi, Emad Salawati, Mohammed Samannodi

**Affiliations:** 1 Department of Pediatrics, Umm Al-Qura University, Makkah, SAU; 2 Internal Medicine, King Fahad Armed Forces Hospital, Jeddah, SAU; 3 College of Medicine, Umm Al-Qura University, Makkah, SAU; 4 Histopathology, King Fahad Armed Forces Hospital, Jeddah, SAU; 5 Department of Pharmacology and Therapeutics, Umm Al-Qura University, Makkah, SAU; 6 College of Dentistry, Umm Al-Qura University, Makkah, SAU; 7 Family Medicine, King Abdulaziz University Faculty of Medicine, Jeddah, SAU; 8 Department of Medicine, Umm Al-Qura University, Makkah, SAU

**Keywords:** disseminated tb, tb, fever, covid-19, tuberculosis

## Abstract

Diagnosis of tuberculosis was affected during the coronavirus disease 2019 (COVID-19) pandemic. Several studies have shown an association between tuberculosis reactivation and COVID-19, but disseminated tuberculosis was rare. We present a case of a 17-year-old male hospitalized due to a fever of unknown origin for two weeks. The patient recovered from COVID-19 five weeks ago, and his nasopharyngeal severe acute respiratory syndrome coronavirus 2 (SARS-CoV-2) polymerase chain reaction (PCR) was negative on current hospitalization. After investigations, diagnosis of disseminated tuberculosis was made by lymph node biopsy and radiological features. The patient was treated with four anti-tuberculosis medications and had a favorable outcome.

## Introduction

Coronavirus disease 2019 (COVID-19), the ongoing pandemic that originated in China in December 2019, is a significant public health threat. More than 100 million cases and 2.3 million deaths worldwide have been reported to the world health organization (WHO) [1].

The global recession due to the COVID-19 pandemic has affected tuberculosis (TB), the infectious disease with the highest mortality rate worldwide, in several ways [2,3]. In 2014, approximately 1.7 billion people were estimated to have latent tuberculosis [4]. Latent TB infection (LTBI) is when an individual infected with *Mycobacterium tuberculosis *has no clinical symptoms of active TB [5]. LTBI can progress to active TB infection in response to bacterial, host, or environmental-related factors [6].

The protective immune response in TB depends mainly on CD4+ T-cells, with the support of CD8+ T-cells. The lack of CD4+ T-cells could increase the susceptibility to tuberculosis [7,8]. A study reported pronounced lymphopenia and a decrease in CD4+ T-cell count in COVID-19 patients [9].

The article "Disseminated Tuberculosis Post COVID-19 Infection: A Case Report" was published in 2022. Journal: Cureus.

Viral infections such as HIV and influenza have been shown to play a role in the reactivation of LTBI [10,11]. Moreover, a recent study suggested that patients with severe COVID-19 could be at higher risk of reactivating latent viral infections such as the Herpes simplex virus [12].

The association between COVID-19 and tuberculosis infection has been reported in several studies that suggested that active or latent TB infection increases the susceptibility to COVID-19 [13]. However, information regarding the role of COVID-19 in the reactivation of LTBI is scarce. We present a case of a young patient initially diagnosed with mild COVID-19, followed by disseminated TB infection in the form of TB lymphadenitis and Pott's disease.

## Case presentation

A 17-year-old male presented to the emergency department with an objective fever of 38°C, fatigue, and a 6 kg weight loss over two weeks. He was diagnosed with mild COVID-19 five weeks before the onset of these symptoms and responded well to supportive treatment.

The patient denied any cough, chest pain, or shortness of breath. There was no history of diarrhea, abdominal pain, vomiting, and urinary symptoms. He is not a smoker and takes no medications. Upon examination, the patient was conscious, alert, ill-appearing, sweating, febrile, and had a temperature of 38.3°C. His blood pressure was 115/85 mmHg, pulse rate was 105 beats per minute, and respiration rate was 20 breaths per minute. The cardiovascular assessment was normal, and the chest had equal bilateral air entry without crepitations or added sounds. The abdomen was soft and lax, and there was no organomegaly or palpable enlarged lymph nodes.

The patient was transferred to the medical unit and admitted for 10 days in order to complete the necessary tests to determine the cause of the high-grade fever. Laboratory investigations were significant for leukocytosis (WBC was 14000x10^9^ cells/liter) and lymphopenia (the absolute lymphocytic count was 800x10^9^ cells/liter). Blood cultures for bacterial growth were negative, as were urine and throat cultures. Nasopharyngeal respiratory multiplex and brucella serology were negative. The echocardiogram was unremarkable.

Computed tomography (CT) of the chest with intravenous (IV) contrast revealed multiple bilateral cervical lymphadenopathies with necrosis, right supraclavicular lymphadenopathy, multiple enlarged mediastinal lymph nodes with central necrosis, and bony lytic lesion in T10 and T12 (Figure 1).

**Figure 1:** CT chest with IV contrast showed bony lytic lesions on T10 and T12 IV: Intravenous

CT abdomen with oral and IV contrast showed multiple enlarged peritoneal lymphadenopathies. Ultrasound-guided lymph node core biopsy of the supraclavicular lymph node revealed multiple caseating granulomas with acid-fast bacilli positivity (Figures 2, 3). Mycobacterial culture of the lymph node biopsy for six weeks was inconclusive.

The article "Disseminated Tuberculosis Post COVID-19 Infection: A Case Report" was published in 2022. Journal: Cureus.

**Figure 2:** Positive AFB stain on supraclavicular lymph node biopsy (H&E, 40×) H&E: Hematoxylin and Eosin; AFB: Acid-fast bacteria

**Figure 3:** Histopathology of supraclavicular lymph node (H&E, 10×). H&E: Hematoxylin and Eosin Histopathology showed caseating granulomata surrounded by epithelioid histiocytes.

Based on the AFB smear of the lymph node and the patient's response to anti-tuberculous treatment, the final diagnosis was disseminated tuberculosis involving the lymph nodes (TB lymphadenitis) and the spine (Pott’s disease). In accordance with the guidelines for initial therapy, the patient was started on four anti-tuberculosis medications for nine months, including oral isoniazid, rifampin, ethambutol, and pyrazinamide. The fever subsided after the initiation of therapy, and the patient had a favorable outcome.

## Discussion

According to the WHO global tuberculosis report 2020, the incidence rate of TB is falling slowly, with a cumulative reduction of 9% (from 142 to 130 new cases per 100 000 population) from 2015 to 2019. Among 54 countries globally, a few Eastern Mediterranean countries, including Saudi Arabia, reported a low TB incidence in 2019. However, it is a significant concern that the COVID-19 pandemic could reverse the recent progress toward TB targets globally [14].

COVID-19 infection has been reported in patients with current or previous TB infection in several studies, including a recent series of 49 cases of COVID-19 and TB co-infection recruited by the Global Tuberculosis Network (GTN) in eight countries, which included 14 patients diagnosed with TB infection shortly after COVID-19 infection [15]. However, they could not detect the role played by COVID-19 in the reactivation of LTBI. Recently, two reports have described the progression of LTBI to active TB following COVID-19 infection; one was reported in Saudi Arabia for an adult patient who had previous contact with a confirmed TB patient two years before mild COVID-19 infection followed by active TB. The author suggested that the reduction of CD4+ T-cell count caused by COVID-19 might have contributed to the reactivation of LTBI [16]. The other case reported the reactivation of TB in a critically ill patient with comorbidities and COVID-19-associated severe acute respiratory distress syndrome (ARDS) who was intubated and started on high-dose steroids with tocilizumab upon his treatment course [17]. However, since steroids and immunosuppressants reduce immune system activity, this patient's development of active TB could not be attributed to COVID-19 only. A study on the implication of COVID-19 on TB has suggested that patients positive for COVID-19 should be screened for LTBI before initiating therapy with immunosuppressive medications and corticosteroids. The WHO even emphasized prescribing a preventive LTBI drug for known positive LTBI cases [18].

The article "Disseminated Tuberculosis Post COVID-19 Infection: A Case Report" was published in 2022. Journal: Cureus.

Our patient is a previously healthy young patient who presented with constitutional symptoms five weeks following mild COVID-19 that did not require the use of immunosuppressive agents or hospitalization. Despite the unremarkable past medical history and the negative purified protein derivative skin (PDD) test result, the unexplained fever and weight loss with the lymphopenia raised the suspicion of TB diagnosis. The involvement of multiple lymph nodes and the lytic lesions at the thoracic spine found on the CT scan with the lymph node biopsy findings confirmed the diagnosis of disseminated TB infection. This could support the association between COVID-19-related immune suppression and the reactivation of TB, suggesting that COVID-19 might accelerate the progression of LTBI to a severe form of TB, even in mildly infected patients. A recent paper has linked lymphopenia during COVID-19 infection to the reactivation of LTB. This is through a process that activates a specific gene stemness, ultimately leading to MTB reproduction and reactivation. However, this phenomenon is yet to be confirmed, as it’s been observed in mice [19].

## Conclusions

This report presented a previously healthy young patient with constitutional symptoms following mild COVID-19. Despite an insignificant medical history and a negative PDD test result, the patient's unexplained fever, weight loss, and lymphopenia prompted a TB diagnosis suspicion. This could support the association between COVID-19-related immune suppression and the reactivation of TB, suggesting that COVID-19 might accelerate the progression of LTBI to a severe form of TB, even in mildly infected patients. Along with the previous reports, it emphasizes the need for further studies to investigate the extent of COVID-19 contribution to the reactivation of LTBI to direct attention to this problem that clearly could increase the burden of TB globally, especially in endemic areas.
